This article has been retracted.

# Value of Biochemical Indexes of Bone Metabolism in Predicting Osteoporotic Lumbar Fractures

**DOI:** 10.1155/2022/7348884

**Published:** 2022-06-23

**Authors:** Fen Feng, CiLa Zhou, Ping Huang, QiaoLin Zhu, Gang Wang, Bin Zhou

**Affiliations:** ^1^School of Pharmacy, Shaoyang University, Shaoyang 422000, China; ^2^Department of Endocrinology, The Central Hospital of Shaoyang, Shaoyang 422000, China

## Abstract

**Objective:**

To investigate the value of bone metabolism indexes such as type I procollagen N-terminal propeptide (P1NP), 25-hydroxyvitamin D (25(OH)D), osteocalcin (OSTEOC), and parathyroid hormone (PTH) in predicting osteoporotic lumbar fractures.

**Methods:**

120 female patients with osteoporosis treated in our hospital were selected as research objects. There were 76 cases in the fracture group and 44 cases in the nonfracture group. The relationship between the levels of P1NP, 25(OH)D, OSTEOC, and PTH and the incidence of osteoporotic lumbar fractures were detected and compared between the two groups. The predictive value of biochemical indexes of bone metabolism in patients with osteoporosis was analyzed by ROC curve.

**Results:**

The levels of P1NP and PTH in the fracture group were significantly higher than those in the nonfracture group, while 25(OH)D and OSTEOC levels were lower than those in the nonfracture group. Moreover, the levels of P1NP, 25(OH)D, OSTEOC, and PTH are important factors affecting the pathogenesis of osteoporosis. The area under the curve (AUC) of fracture in patients with osteoporosis predicted by the combination of P1NP, 25(OH)D, OSTEOC, and PTH levels was 0.886, which was greater than the AUC predicted by each index (0.796, 0.753, 0.670, and 0.824). The best sensitivity and specificity of comprehensive prediction of each index were 78.95% and 79.10%, respectively.

**Conclusion:**

The abnormal changes of P1NP, 25(OH)D, OSTEOC, and PTH in female patients with osteoporotic lumbar fracture are closely related to the occurrence of the disease. The combination of these indicators has relatively significant application value in predicting the occurrence of fracture, which is helpful to formulate and guide relevant preventive measures for female patients with osteoporotic lumbar fracture and improve the prognosis.

## 1. Introduction

Osteoporotic fractures are mainly caused by primary osteoporosis, which results in a decrease in bone density and bone quality, thus leading to a decrease in bone strength [1]. Once impacted by an external force, a patient with primary osteoporosis may suffer a fracture. Therefore, primary osteoporosis has become a main cause of fractures and disability in the elderly [2]. At present, clinical diagnosis of osteoporosis is mainly based on the bone mineral density (BMD) examination [3]. Older women with osteoporosis have lower BMD and are more likely to have fractures [4]. However, due to certain factors, such as the age of a patient, the accuracy of biochemical indexes of bone metabolism in predicting osteoporosis has been into question [5]. Therefore, the relationship between future bone loss and bone turnover in a patient's body is reflected through clinical dynamic monitoring of biochemical indexes of bone metabolism, which can be used as an important auxiliary method in imageological examinations to predict the risk of osteoporotic lumbar fractures [6]. On this basis, in this study, the clinical data of patients with osteoporosis admitted to the Department of Orthopedics and Traumatology of this hospital was selected and used to observe the correlation between changes in the biochemical indexes of bone metabolism and osteoporosis, which is reported as follows.

## 2. Methods

### 2.1. General Information

A retrospective analysis was carried out on 120 female patients with osteoporosis admitted to this hospital during the period from May 2018 to January 2020.

The following are the inclusion criteria: (1) DXA measurement and *T*-score that meet the diagnostic criteria of osteoporosis (≤-2.5SD) for the hip and lumbar spine [7]; (2) no surgery, hormone drugs, vitamin D, parathyroid hormone, or other similar treatments before enrollment; (3) no thyroid disease; and (4) patients or their families who signed an informed consent. The following are the exclusion criteria: (1) patients have hemopathy; (2) patients have diabetes, rheumatism, any immune diseases, Cushing's syndrome, etc.; (3) patients have malignant tumor; (4) patients have serious infectious diseases; (5) patients have serious cardiovascular and cerebrovascular diseases and liver and kidney dysfunction; 6) patients have any built-in objects for joint replacement or lumbar surgery; and (7) patients have fractures caused by accidental injuries.

According to the occurrence of lumbar fracture after osteoporosis, the patients were divided into the fracture group (*n* = 76) and the nonfracture group (*n* = 44). This study was approved by the Medical Ethics Committee of Shaoyang Central Hospital.

### 2.2. Biochemical Detection

In the fracture group, 5 ml of fasting venous blood was collected in the early morning after admission. For the nonfracture group, 5 ml of fasting venous blood was collected during physical examination. Blood samples were then centrifuged at 3500 r/min for 5 minutes to collect serum and stored at -80°C. The N-terminal propeptide (P1NP) of type I procollagen was detected by the o-cresol phthalein complexing agent method. Professional testers were used electrochemiluminescence to detect serum 25(OH)D, osteocalcin (OSTEOC), and parathyroid hormone (PTH). The 25(OH)D kit, OSTEOC kit, and PTH kit were purchased from Roche Diagnostics (Shanghai) Co., Ltd. (China). The test was carried out in strict accordance with the instructions of the kits.

### 2.3. Statistical Analysis

The data was processed by SPSS22.0 software. The measured data was expressed as the mean ± standard deviation (SD) and analyzed using a *t*-test. The count data is expressed in *n* (%) and compared using the *χ*^2^ test. Multiple regression analysis was logistic regression analysis. The predicted values were analyzed by the receiver operating characteristic (ROC) curve. When *P* < 0.05, the difference was statistically significant.

## 3. Results

### 3.1. General Information and BMD Data of the Two Groups

The basic information of the patients is shown in Table 1. The 120 patients included were aged 55-78 years, with an average age of 59.2 ± 75.52 years. Their body mass ranged from 67 to 85 kg, and the average body mass was 62.09 ± 5.37 kg. There was no significant difference in age, body weight, and body mass index between the two groups (*P* > 0.05).

In addition, there was no statistically significant difference in the BMD of the lumbar vertebrae and the hip between the two groups (*P* > 0.05) (Table 2).

### 3.2. Biochemical Indexes of Bone Metabolism of the Two Groups

We further analyzed the bone metabolic indexes in the serum of patients in the two groups. The 25(OH)D and OSTEOC levels of the fracture group were lower than those of the nonfracture group (*P* < 0.05). And the P1NP and PTH levels in the fracture group were significantly higher than in the nonfracture group (*P* < 0.05) (Table 3).

### 3.3. The Relationship between Biochemical Indexes of Bone Metabolism and the Incidence of Osteoporotic Lumbar Fractures

Furthermore, logistic regression analysis showed that P1NP (OR = 4.954; 95%CI : 2.748 − 8.931; *P* < 0.001), 25(OH)D (OR = 3.340; 95%CI : 1.908 − 5.846; *P* < 0.001), and OSTEOC (OR = 5.613; 95%CI : 3.569 − 8.827; *P* < 0.001) were risk factors for the incidence rate of lumbar osteoporosis. However, PTH (OR = 0.430; 95%CI : 0.272 ~ 0.680; *P* < 0.001) was a protective factor affecting the incidence rate of lumbar osteoporosis (Table 4).

### 3.4. ROC Curves of Biochemical Indexes of Bone Metabolism in Patients with Osteoporotic Lumbar Fractures

Finally, we used ROC curves to determine the accuracy of bone metabolic indexes as a diagnosis tool for the occurrence of osteoporotic fractures. The result (Figure 1) showed that, for P1NP of the lumbar vertebrae, the area under the curve (AUC) was 0.796 (*P* < 0.05), the 95% CI was 0.696~0.875, the cut-off value was ≤88.87, and the corresponding sensitivity and specificity of prediction were 78.95% and 73.13%, respectively; for serum 25(OH)D, the AUC was 0.753 (*P* < 0.05), the 95% CI was 0.649~0.840, the cutoff value was ≤13.35 ng/ml, and the corresponding sensitivity and specificity of prediction were 84.21% and 59.70%, respectively; for OSTEOC (BGP), the AUC was 0.670 (*P* < 0.05), the 95% CI was 0.560~0.767, the cutoff value was ≤7.68 ng/ml, and the corresponding sensitivity and specificity of prediction were 63.16% and 73.13%, respectively; for PTH, the AUC was 0.824 (*P* < 0.05), the 95% CI was 0.727~0.898, the cutoff value was >40.62 pmol/L, and the corresponding sensitivity and specificity of prediction were 78.95% and 74.63%, respectively; for the combination of the indexes, the AUC was 0.886 (*P* < 0.05), the 95% CI was 0.799~0.945, the *Z*-score was 9.319, and the best sensitivity and specificity of were 78.95% and 79.10%, respectively.

## 4. Discussion

With the accelerated aging of the population in China, the incidence of osteoporosis has increased year by year [8]. In recent years, in-depth studies on the pathogenesis of osteoporosis and continuous improvement in treatment methods have led to a significant improvement in the results of clinical treatment of osteoporosis. However, the early symptoms of osteoporosis are clinically insignificant or even nonspecific, seriously affecting clinical diagnosis and treatment of the disease [9, 10]. In this study, no significant difference in the BMD of the hip and lumbar vertebrae was found between the fracture group and the nonfracture group. However, the BMD of the lumbar vertebrae was higher than that of the hip, which might be the result of hyperostosis caused by lumbar degeneration. So vertebral compression fracture was selected as the object of this study.

Imageological examination is the most preferred method for clinical evaluation of osteoporosis [11]. Dual-energy X-ray absorptiometry can be used to comprehensively evaluate the BMD of the lumbar vertebrae and the hip joint, which has obvious advantages, especially in the accuracy of BMD for two-dimensional planes of different bones (the sum of cortical bone and cancellous bone). However, it cannot measure the cortical bone and the cancellous bone separately, resulting in a relatively large error in the measurement of the actual bone content in the cancellous bone, which affects its application effect [12]. Clinical studies confirmed [13] that abnormal expression and examination of biomarkers of bone metabolism can reflect the BMD of patients, which can be used as important indexes for predicting osteoporosis. Moreover, studies have showed that markers of bone metabolism are secreted by osteoblasts or osteoclasts, so various indexes of bone metabolism are better than BMD in evaluating the progress of each stage of osteoporosis [14]. Therefore, monitoring changes in the biochemical indexes of bone metabolism is of great significance for predicting osteoporotic fractures. Krege et al. showed that an increase in the P1NP level reflects the accelerated synthesis of type I collagen, indicating active bone turnover [15]. Studies [16, 17] confirmed that lack of vitamin D is an important factor in the occurrence and development of osteoporosis, and 25(OH)D is a sensitive index reflecting the nutritional status of vitamin D in the body. Therefore, detection of serum 25(OH)D is helpful for the diagnosis and evaluation of osteoporosis. And changes in the P1NP level are closely related to the occurrence of postmenopausal osteoporotic lumbar fractures [18]. In addition, some clinical studies [19, 20] also showed that the expression of serum OSTEOC in patients with osteoporosis was significantly reduced, while the level of PTH was abnormally increased, which was closely related to the occurrence and development of the disease. The results of this study demonstrated that the levels of P1NP and PTH of the fracture group were higher than those of the nonfracture group, while the levels of 25(OH)D and OSTEOC of the fracture group were significantly lower than those of the nonfracture group, which were consistent with the results of the aforementioned studies. It was found through the logistic regression analysis in this study that levels of P1NP, serum 25(OH)D, OSTEOC, and PTH are important factors affecting the incidence of osteoporotic lumbar fractures. This study indicated that after some influencing factors, such as patient age and gender, were excluded, the above indexes were still significantly related to the occurrence of osteoporosis, fully demonstrating that changes in the levels of these indexes were involved in the occurrence and development of osteoporosis. What is more, in this study, the value of the above indexes in the assessment of the risk of fractures in patients with osteoporosis was analyzed with ROC curves, indicating that the AUC of the combination of the biochemical indexes of bone metabolism in predicting fractures in patients with osteoporosis was up to 0.886, and the best sensitivity and specificity of prediction were 78.95% and 79.10%, respectively, which can basically meet the requirements of prediction and provide important references for the clinical assessment of prognosis in patients. However, if it is required that the sensitivity must be greater than 90%, the specificity will be significantly reduced, and the misdiagnosis rate will increase.

To sum up, there is a significant correlation between osteoporotic lumbar fractures and abnormal expression of the levels of P1NP, PTH, 25(OH)D, and OSTEOC. The combination of the above indexes helps doctors evaluate the risk of osteoporotic lumbar fractures and has a significant clinical application value. However, further studies with larger sample sizes are required to determine the threshold of each index in assessing the degree of osteoporosis and risk of fractures.

## Figures and Tables

**Figure 1:** ROC curves of the biochemical indexes of bone metabolism for prediction.

**Table 1:** Comparison of general information between the two groups.

Variable	Fracture group (*n* = 76)	Nonfracture group (*n* = 44)	*t*	*P*
Age (years old)	58.56 ± 6.17	59.27 ± 5.52	0.795	0.428
Body mass (kg)	61.82 ± 4.85	62.09 ± 5.37	0.346	0.730
BMI (kg/m^2^)	27.35 ± 5.75	26.68 ± 5.84	0.845	0.358

Data was expressed as the mean ± standard deviation (SD). BMI: body mass index.

**Table 2:** Comparison of biochemical indexes of bone metabolism between the two groups.

Variable	Fracture group (*n* = 76)	Nonfracture group (*n* = 44)	*t*	*P*
BMD of the lumbar vertebrae (g/cm^2^)	0.61 ± 0.04	0.60 ± 0.05	1.583	0.089
BMD of the hip (g/cm^2^)	0.69 ± 0.04	0.68 ± 0.05	1.353	0.940

Data was expressed as the mean ± SD. BMD: bone mineral density.

**Table 3:** Comparison of biochemical indexes of bone metabolism between the two groups.

Variable	Fracture group (*n* = 76)	Nonfracture group (*n* = 44)	*t*	*P*
P1NP (ng/ml)	66.82 ± 20.04	49.54 ± 15.27	-16.803	<0.001
25(OH)D3 (ng/ml)	13.58 ± 3.21	20.39 ± 3.74	12.814	<0.001
OSTEOC (ng/ml)	8.05 ± 1.96	13.84 ± 3.52	13.327	<0.001
PTH (pmol/l)	39.02 ± 6.28	18.63 ± 5.50	22.651	<0.001

Data was expressed as the mean ± SD.

**Table 4:** Relationship between biochemical indexes of bone metabolism and incidence of osteoporotic lumbar fractures.

Variate	*β*	S.E.	Wald *χ*^2^	*P*	OR	95% CI
P1NP	1.600	0.491	10.622	<0.001	4.954	2.748~8.931
25(OH)D	1.206	0.405	8.866	<0.001	3.340	1.908~5.846
OSTEOC	1.725	0.560	9.489	<0.001	5.613	3.569~8.827
PTH	-0.844	0.261	10.452	<0.001	0.430	0.272~0.680

## Data Availability

The data used to support the findings of this study are available from the corresponding author upon request.
